The article "Clinical Efficacy of Interventional Therapy on Lower Extremity Arteriosclerosis Obliterans and Prognostic Factors" was retracted in 2023. Reasons: unreliable results or conclusions; lack of ethics approval or compliance; concerns about the data; concerns about the peer review.

# Clinical Efficacy of Interventional Therapy on Lower Extremity Arteriosclerosis Obliterans and Prognostic Factors

**DOI:** 10.1155/2022/9190292

**Published:** 2022-08-04

**Authors:** Deshuang Xiao, Jun Song

**Affiliations:** General Surgery, The First People's Hospital of WenLing, No. 333, Chuanan Road, Wenling City, 317500 Zhejiang Province, China

## Abstract

**Objective:**

This study was designed to analyse the clinical efficacy of interventional therapy on lower extremity arteriosclerosis obliterans (LEASO) and prognostic factors.

**Methods:**

A total of 122 patients with LEASO diagnosed in our hospital from March 2017 to March 2019 were retrospectively analysed. Among them, 72 patients who received conservative therapy were assigned to a conservative group, and 50 patients who received interventional therapy additionally based on conservative therapy were assigned to an intervention group. The short-term (12 weeks after therapy) and long-term (3 years after therapy) clinical efficacies on the two groups were compared. Death, amputation, and vascular restenosis (vascular stenosis > 50% in computed tomography reexamination) were defined as unfavourable outcomes, and Cox regression was conducted to analyze the factors influencing the prognosis of patients. The incidence of adverse events in the two groups within 3 years was compared and statistically analyzed. Additionally, the hospital stay, therapy cost, claudication distance, and ankle brachial index were compared between the two groups.

**Results:**

After therapy, the conservative group showed a notably lower total effective rate than the intervention group (*P* < 0.05), but the clinical efficacy after 3 years was similar between the two groups (*P* > 0.05). Additionally, the conservative group experienced notably longer hospital stay than the intervention group (*P* < 0.05), and cost less in treatment than the intervention group (*P* < 0.05). However, the conservative group experienced a notably shorter claudication distance and showed a notably lower ankle brachial index than the intervention group (*P* < 0.05). The two groups were not significantly different in mortality, amputation rate, and vascular restenosis rate (*P* > 0.05). Moreover, Cox regression analysis revealed that age and conservative therapy were independent risk factors for the prognosis of patients (*P* < 0.05).

**Conclusion:**

Interventional therapy can substantially improve the short-term efficacy and prognosis of patients with LEASO, but the cost is high, so the therapeutic regimen should be selected according to the patient's economic condition.

## 1. Introduction

Peripheral arterial disease (PAD) is a common vascular disease [1, 2]. Lower extremity arteriosclerosis obliterans (LEASO), as a kind of PAD, is a chronic progressive disease [3]. Arterial stenosis and occlusion triggered by arterial intimal thickening and atherosclerosis give rise to limb blood supply insufficiency, resulting in a series of symptoms and signs of the affected limb [4]. According to recent research, with the development of society, the improvement of living standards, and the trend of aging, the prevalence of LEASO is increasing [5]. Surveys show that the incidence of peripheral arterial ischemic disease among people over 70 years old is approximately 15%-20% in western countries, while it reaches 15.91% in China [6, 7]. Not only that, limb ischemia triggered by LEASO causes a soaring disability and mortality, which seriously worsens the prognosis of patients [8].

The therapy methods of LEASO mainly include general therapy, drug therapy, traditional surgical therapy, and percutaneous endovascular therapy [9]. Over the past few years, many new methods such as hybrid surgery, stem cell transplantation, and laser-assisted angioplasty have been adopted in clinical practice to varying degrees [10]. At the current stage, surgery and interventional therapy are effective in relieving arterial occlusion [10]. Interventional therapy is a frequently adopted therapy method for patients with LEASO, with characteristics of simple operation, little trauma, and high safety [11]. However, its long-term efficacy is still under controversial [12]. Therefore, it is of great significance to design scientific and standardized perioperative nursing interventions to improve the therapy effect, reduce the risk of complications, and improve the therapy services.

This study was designed to analyze the clinical efficacy of interventional therapy on LEASO and prognostic factors to provide reference for clinical therapy.

## 2. Methods and Data

### 2.1. Clinical Data of Patients with LEASO

A total of 122 patients with LEASO diagnosed in our hospital from March 2017 to March 2019 were retrospectively analysed. Among them, 72 patients who received conservative therapy were assigned to a conservative group (Con group), and 50 patients who received interventional therapy additionally based on conservative therapy were assigned to an intervention group. This study was ratified and approved by the Medical Ethics Committee of our hospital.

### 2.2. Inclusion and Exclusion Criteria

The inclusive criteria are as follows: patients with intermittent claudication of lower limbs, patients with ankle brachial index (ABI) < 0.9, patients whose results of color Doppler ultrasound or computed tomography angiography of lower limb artery indicated that the stenosis degree of diseased artery lumen was ≥50%, patients who met the diagnostic criteria proposed by the Vascular Surgery Branch of Surgery Society of Chinese Medical Association in 2015 [13], and those with detailed clinical data.

The exclusion criteria are as follows: patients with malignant tumour, patients with dysfunction in the liver, kidney, or other important organs, patients with coagulation dysfunction, and those with schizophrenia, depression, or other mental disorders.

### 2.3. Therapeutic Regimen

The conservative group was given conservative therapy as follows: general drug therapy: each patient was required to keep good living habits such as quitting smoking and drinking, light diet, regular work, and rest. Staff were arranged to control the blood pressure, blood lipid, and blood glucose of each patient, and patients suffering from chronic diseases such as heart disease, lung disease, and kidney disease should be given appropriate medication, and those with lower extremity arterial diseases were given aspirin or clopidogrel-monoclonal antibody. Exercise therapy: the staff instructed the patients to go outside the hospital before discharge in the premise of ensuring safety. The suggested training methods included walking, stretching, and bending ankles. Each patient was recommended to walk for 30-45 minutes each time (it can be gradually increased according to ischemic symptoms), and patients without ischemic symptoms were recommended to walk at least 3 times a week for at least 12 weeks.

The intervention group was given interventional therapy: balloon dilatation or stent implantation was performed on the basis of conservative therapy. Each patient was let to lie in a horizontal position. After successful local anesthesia, the contralateral femoral artery or left arm artery was punctured, and a catheter sheath was inserted. After the lesion was identified by angiography, the sheath was replaced with a long sheath. Then, the patient was injected intravenously with 30-50 mg heparin. The guide wire was used with the catheter together to guide normal and/or drug-coated balloons pass through narrow and/or occluded lethal arterial incisions. If the stenosis was still more than 30%, or local arterial dissection was formed after balloon expansion, a stent was placed. For the stenosis or occlusion of the inferior genicular artery, a balloon with the diameter equal to that of the blood vessel or slightly smaller than it was selected for expansion and shaping according to the diameter of the diseased blood vessel to ensure that there was at least one outlet channel under the knee, followed by opening. Anticoagulant drugs (oral rivaroxaban) were given on the basis of long-term conservative therapy after operation for at least 12 weeks.

### 2.4. Outcome Measures

Primary observation indexes: the short-term (12 weeks after therapy) and long-term (3 years after treatment) clinical efficacies on the two groups were compared; clinical evaluation criteria: markedly effective: computed tomography angiography or angiography showed stenosis < 30%, symptom disappearance, and no serious complications. Effective: angiography showed stenosis < 50%, symptom alleviation, and no serious complications; ineffective: no symptom alleviation and no symptom aggravation; deteriorated: vascular stenosis > 70% and worse symptoms. The total effective rate = markedly effective rate + effective rate [14]. The incidence of adverse events in the two groups within 3 years was compared and statistically analyzed. Death, amputation, and vascular restenosis (vascular stenosis > 50% in computed tomography reexamination) were defined as unfavourable outcomes, and Cox regression was conducted to analyse the factors influencing the prognosis of patients.

Secondary outcome measures: the clinical data between the two groups were compared. The incidence of adverse events in the two groups within 3 years was compared and statistically analyzed. Additionally, the two groups were compared in hospital stay, therapy cost, claudication distance, and ABI.

### 2.5. Statistical Analyses

SPSS20.00 software was used for analysis of the collected data, and GraphPad Prism 8 software was adopted for visualization of the data into corresponding figures. Counting data were compared using the chi-square test, and measurement data were compared between groups using the independent *t* test and compared within groups before and after therapy using the paired *t* test. Cox regression was conducted to analyse the independent prognostic factors. *P* < 0.05 implies a statistically significant difference.

## 3. Results

### 3.1. Baseline Data of Patients

According to comparison of baseline data between the conservative group and intervention group, there was no significant difference between the two groups in age, sex, course of disease, history of smoking, history of hypertension, history of diabetes, and history of coronary heart disease (*P* > 0.05, Table 1).

### 3.2. Clinical Efficacy Analysis

According to comparison of the two groups in clinical efficacy after therapy and 3 years of therapy, the conservative group showed a significantly lower total effective rate than the intervention group after therapy (*P* < 0.05, Table 2), but further comparison revealed that there was no significant difference between them in clinical efficacy after 3 years of therapy (*P* > 0.05, Table 3).

### 3.3. Changes of Rutherford Grading in Patients before and after Therapy

The Rutherford grades of the two groups before and after therapy were compared. According to the results, the two groups were not significantly different in Rutherford grading before therapy (*P* > 0.05, Table 4), but after therapy, the intervention group had a notably lower proportion of patients with grade 4-6 than the conservative group (*P* < 0.05, Table 4).

### 3.4. Comparison of Hospital Stay, Therapy Cost, Claudication Distance, and ABI

The two groups were compared in hospital stay, therapy cost, claudication distance, and ABI. The conservative group experienced notably longer hospital stay than the intervention group (*P* < 0.05, Figure 1(a)), and cost less in therapy than the intervention group (*P* < 0.05, Figure 1(b)). Additionally, the conservative group experienced notably lower claudication distance and showed a notably lower ABI than the intervention group (*P* < 0.05, Figures 1(c) and 1(d)).

### 3.5. Incidence of Adverse Events

The incidence of adverse events in the two groups during 3 years after therapy was statistically analyzed, and the two groups were found to be not significantly different in mortality, amputation rate, and vascular restenosis rate (*P* > 0.05, Table 5).

### 3.6. Analysis of Prognostic Factors of Patients

According to the occurrence of adverse events in 3 years, the patients were assigned to the favourable-prognosis group or an unfavourable-prognosis group. Their clinical data were collected and assigned (Table 6). Univariate Cox regression analysis showed that age, course of disease, and therapeutic regimen were correlated with prognosis (*P* < 0.05, Table 7). Further analysis showed that age and conservative therapy were independent risk factors affecting the prognosis of patients (*P* < 0.05, Table 7), and patients with advanced age, long course of disease, and conservative therapy showed a notably lower survival rate than those with younger age, short course of disease, and combined interventional therapy (*P* < 0.05, Figure 2).

## 4. Discussion

LEASO is refractory, and its prognosis is unfavourable. Although conservative therapy can improve patients' microcirculation and fight against infection, it has not achieved ideal results for LEASO [15]. In recent years, with the improvement of medical level and medical instruments, interventional therapy is extensively applied because of its minimal invasion, safety, good curative effect, and easy recovery [16]. Thrombolysis, balloon dilatation, intracavitary rotary cutting, stent implantation, artery dilatation, and reconstruction are commonly used interventional therapy methods [17]. Interventional therapy has become the first choice for LEASO. In recent years, thanks to the improvement of technology and equipment, the interventional therapy of LEASO has made remarkable progress, and the success rate and short-term efficacy of it after operation have been lifted [18].

In this study, the efficacy of conservative therapy and interventional therapy on patients with LEASO were compared, and notably, better clinical efficacy on patients given interventional therapy was found than that on patients given conservative therapy. However, there was no significant difference in clinical effective rate between the two groups after 3 years. This shows that interventional therapy can substantially improve the short-term efficacy, without significant effect on the long-term efficacy on patients with LEASO. Moreover, analysis in the present study also found that patients in the conservative group experienced longer hospital stay, cost less in therapy, experienced a shorter claudication distance, and showed a lower ABI compared with the intervention group. The Rutherford grades of patients were compared, and a notably smaller number of patients with Rutherford grades 4-6 was found in the intervention group than that in the conservative group after therapy. The results suggest that interventional therapy can effectively expand and reconstruct the narrow or even occluded blood vessels of patients, improve the blood circulation, and thus, significantly increase the patency rate of blood vessels, reduce Rutherford grade, and increase the claudication distance and ABI, significantly improving the total effective rate [12, 19]. Although conservative therapy can improve the microcirculation of patients, it exerted a slow effect and prolonged hospital stay [20]. However, the cost of interventional therapy is greatly increased due to the use of consumables. Therefore, the therapy should be selected according to the patient's own economic conditions.

The continuous development of medical devices in recent years has lowered the mortality and amputation rate of patients with LEASO [21]. However, some data show that there are still some adverse events such as cardiovascular and cerebrovascular diseases, amputation, and death [22]. LEASO, as a systemic disease, is often complicated with many diseases, such as hypertension, diabetes, ulcer, and gangrene in severe lower limb ischemia, which may lead to amputation, and the aggravation of complications may result in death [23]. The incidence of adverse events in the two groups within three years was counted, and no difference was found in death, amputation, and restenosis between them. Moreover, the patients were further grouped according to adverse events. Through Cox regression analysis, conservative therapy and age ≥ 70 years were found to be independent risk factors affecting the prognosis of LEASO. According to research, the incidence of LEASO increases with the increase of age, and the incidence of it among people over 70 years old is significantly higher than that among people under 70 years old [24]. Moreover, it was found that the probability of unfavourable prognosis among patients over 70 years old was 2.206 times than that among patients under 70 years. The results indicate that the older the patient is, the higher the probability of unfavourable prognosis is. We also found that patients given conservative therapy showed a higher probability of unfavourable prognosis than those given interventional therapy, indicating notable better clinical effect and prognosis of interventional therapy than conservative therapy [25]. Therefore, during therapy of patients with LEASO, attention should be paid to age, and elderly patients should be given interventional therapy to ensure their prognosis.

This study has confirmed that interventional therapy has a significant short-term effect in patients with LEASO and can substantially improve the prognosis of patients, but it still has some limitations. First of all, the sample size in this study is small. Secondly, this study, as a retrospective study, cannot follow up the patients for a long time like a prospective study. In this study, we checked the outpatient review records to count the adverse outcomes of patients, but did not count the outcomes of patients without reexamination. Therefore, we hope to carry out prospective research, with a larger sample size and a long-term follow-up in the future to improve our conclusion.

To sum up, interventional therapy can substantially improve the short-term efficacy and prognosis of patients with LEASO, which is worthy of clinical promotion.

## Figures and Tables

**Figure 1:** Comparison of hospital stay, therapy cost, claudication distance, and ankle brachial index. (a) Comparison of hospital stay between the two groups after therapy; (b) comparison of the therapy cost between the two groups after therapy; (c) comparison of claudication distance between the two groups after therapy. (d) Comparison of ankle brachial index between the two groups after therapy. Note: ^∗∗∗^*P* < 0.001.

**Figure 2:** *K*-*M* curve of unfavourable prognosis of patients with different age, course of disease, and therapeutic regimens. (a) *K*-*M* curve of unfavourable prognosis of patients aged ≥70 and those <70; (b) *K*-*M* curve of unfavourable prognosis of patients with course of disease ≥4 years and those with course of disease <4 years; (c) *K*-*M* curve of unfavourable prognosis of patients given conservative therapy and those given interventional therapy.

**Table 1:** Comparison of baseline data between the conservative group and intervention group.

Items		Conservative group (*n* = 72)	Intervention group (*n* = 50)	*P* value
Age (years)		70.30 ± 6.17	69.44 ± 5.81	0.437
Gender				0.223
	Male	44	25	
	Female	28	25	
Course of disease (years)		3.89 ± 0.64	4.00 ± 0.57	0.3269
History of smoking				0.169
	Yes	45	25	
	No	27	25	
History of hypertension				0.917
	Yes	41	28	
	No	31	22	
History of diabetes				0.359
	Yes	23	20	
	No	49	30	
History of coronary heart disease				0.615
	Yes	37	28	
	No	35	22	

**Table 2:** Comparison of clinical efficacy between the two groups after therapy.

Group	Markedly effective	Effective	Ineffective	Total effective rate
Conservative group (*n* = 72)	10	32	30	58.33%
Intervention group (*n* = 50)	18	23	9	82.00%
*χ* ^2^ value				7.600
*P* value				0.006

**Table 3:** Comparison of clinical efficacy between two groups after 3 years of therapy.

Group	Markedly effective	Effective	Ineffective	Deteriorated	Total effective rate
Conservative group (*n* = 72)	20	19	22	11	54.17%
Intervention group (*n* = 50)	18	12	15	5	60.00%
*χ* ^2^ value					0.408
*P* value					0.523

**Table 4:** Changes of Rutherford grading in the two groups before and after therapy.

Group	Before therapy		After therapy	
	1-3	4-6	1-3	4-6
Conservative group (*n* = 72)	32	40	54	18
Intervention group (*n* = 50)	25	25	45	5
*χ* ^2^ value	0.366		4.340	
*P* value	0.545		0.037	

**Table 5:** Incidence of adverse events in the two groups.

Group	Died	Amputation	Vascular restenosis
Conservative group (*n* = 72)	9	10	9
Intervention group (*n* = 50)	3	3	2
*χ* ^2^ value	1.406	1.929	2.599
*P* value	0.235	0.165	0.107

**Table 6:** Assignment of prognostic factors in the two groups.

Items	Assignment
Age	≥70 years old = 1, <70 years old = 0
Gender	Male = 1, female = 0
Course of disease	≥4 years = 1, <4 years = 0
History of smoking	Yes = 1, no = 0
History of hypertension	Yes = 1, no = 0
History of diabetes	Yes = 1, no = 0
History of coronary heart disease	Yes = 1, no = 0
Therapeutic regimen	Conservative therapy = 1, combined interventional therapy = 0

**Table 7:** Univariate and multivariate Cox regression analysis of the two groups.

Items	Univariate Cox regression			Multivariate Cox regression		
	*P* value	HR value	95% CI	*P* value	HR value	95% CI
Age	0.007	2.612	1.306-5.226	0.028	2.205	1.087-4.472
Gender	0.213	0.660	0.343-1.270			
Course of disease	0.041	2.060	1.030-4.120	0.250	1.518	0.745-3.092
History of smoking	0.816	1.082	0.558-2.099			
History of hypertension	0.317	1.415	0.717-2.794			
History of diabetes	0.645	1.171	0.599-2.288			
History of coronary heart disease	0.281	1.446	0.740-2.825			
Therapeutic regimen	0.011	2.758	1.256-6.056	0.042	2.298	1.030-5.125

Notes: HR: hazard ratio; CI: confidence interval.

## Data Availability

The data used to support the findings of this study are included within the article.
